# m6A RNA Methylation Regulators Contribute to Predict and as a Therapy Target of Pulmonary Fibrosis

**DOI:** 10.1155/2022/2425065

**Published:** 2022-04-21

**Authors:** Meng-Sheng Deng, Kui-Jun Chen, Dong-Dong zhang, Guan-Hua Li, Chang-Mei Weng, Jian-Min Wang

**Affiliations:** State Key Laboratory of Trauma, Burn and Combined Injury, Daping Hospital, Army Medical University, Chongqing 400042, China

## Abstract

**Background:**

Pulmonary fibrosis is difficult to treat. Early diagnosis and finding potential drug therapy targets of pulmonary fibrosis are particularly important. There were still various problems with existing pulmonary fibrosis markers, so it is particularly important to find new biomarkers and drug treatment targets. m6A (N6,2′-O-dimethyladenosine) RNA methylation was the cause of many diseases, and it is regulated by m6A methylation regulators. So, whether RNA methylation regulators can be a diagnostic marker and potential drug therapy target of early pulmonary fibrosis needs to be explored.

**Materials and Methods:**

Using GSE110147 and GSE33566 in the GEO database to predict the m6A methylation regulators that may be related to the development of pulmonary fibrosis, we used 10 mg/ml bleomycin to induce mouse pulmonary fibrosis models and human pulmonary fibrosis samples, to confirm whether this indicator can be an early diagnostic marker of pulmonary fibrosis.

**Results:**

According to the database prediction results, METTL3 can predict the occurrence and development of pulmonary fibrosis, and the results of MASSON and HE staining show that the fibrosis model of mice is successful, and the fibrosis of human samples is obvious. The results of immunohistochemistry showed that the expression of METTL3 was significantly reduced in pulmonary fibrosis.

**Conclusions:**

The m6A methylation regulator METTL3 can be considered as an important biomarker for diagnosing pulmonary fibrosis occurrence, furthermore it could be considered as a drug target because of its low expression in pulmonary fibrosis.

## 1. Introduction

The RNA modification was so ordinary in nature, in almost all types of cellular and all species, N6,2′-O-dimethyladenosine could been found [1, 2]. The m6A modification was the most studied mRNA modification mode. Methyltransferases, blinding proteins, and demethylases play the major roles in RNA methylation modification [3, 4]. The m6A methylation regulators consist of methyltransferases, blinding proteins, and demethylases. At present, methyltransferases contain METTL3 [5], METTL14 [6], RBM15 [7], WTAP [8], ZCH13 [9], KIAA1429 [10], HNRNPC [11], and blinding proteins include YTHDC2 [12], YTHDC1 [13], YTHDF1 [14], YTHDF2 [14], and demethylases have two proteins: FTO and ALKBH5 [9, 12]. m6A modification plays a key role in biological development and disease occurrence. More and more evidence shows that the m6A methylation regulator expression level is related to certain diseases, including fibrosis, tumors, and others [15–17].

The m(6)A methyltransferase methyltransferase-like 3 (METTL3) was shown to be the main methyltransferase of the m(6)A modification on MALAT1. Li et al. [18] and Liu et al. [19] showed that the dihydroartemisinic (DHA) on TGF-beta1-induced renal fibrosis was affected by the MALAT1/miR-145/FAK pathway in vitro and in vivo. It is confirmed that m(6)A modification has functional importance in renal interstitial fibrosis during obstructive nephropathy and might be a promising therapeutic target. To the best of our knowledge, pulmonary fibrosis with molecular markers and clinicopathological characteristics was connected with the expression of m6A methylation regulators in comprehensive analysis [20]. Therefore, mRNA methylation regulators may be a new and reliable predictor of pulmonary fibrosis and a potential drug therapy target.

In our study, the GEO data sets which contain 123 peripheral blood samples has been analyzed systematically which the expression of 10 commonly reported m6A methylation regulators. The relationship between the expression of the m6A methylation regulator and clinicopathological characteristics was also investigated. The expression of m6A methylation regulators can be regarded as important in predicting the clinicopathological characteristics and molecular markers of pulmonary fibrosis. A signature constructed m6A methylation regulators METTL3 might be the diagnosis biomarker and drug target of pulmonary fibrosis in this study.

## 2. Methods

### 2.1. Data Handling

The RNA-seq transcriptome data were downloaded from the GEO database, the data number were GSE110147 and GSE33566 (http://cancergenome.nih.gov/). To normalize the sequencing data downloaded from the GEO database, the expectation‐maximization method was used. The dataset GSE33566 was collected on Agilent microarrays and gene expression profiles of peripheral blood RNA from 93 IPF patients. The dataset GSE110147 was collected by Affymetrix microarrays. The fresh frozen lung samples were obtained from the recipients' organs of 22 patients with IPF, 10 with NSIP, and 5 with mixed IPF-NSIP undergoing lung transplantation.

### 2.2. m6A Methylation Regulators Selection

The 10 m6A methylation regulators in this paper were selected according to references. The expression of these m6A methylation regulators in pulmonary fibrosis with different clinicopathological characteristics was compared.

### 2.3. Bioinformatic Analysis

ConsensusClusterPlus (http://www.bioconductor.org/) was used to cluster separate groups in pulmonary fibrosis data, and 50 iterations, a resample rate of 80%, and the Pearson correlation were used. The expression patterns in different cluster groups were analysed by PCA. The protein-protein interaction analysis was carried out by an online dataset, the STRING database (http://www.string‐db.org/). To evaluate the predictive efficiency of the risk scores, the receiver operating characteristic (ROC) curve was used.

### 2.4. Animal Experiment and Human Sample

A pulmonary fibrosis model was constructed through Bleomycin (BLM). The 6-week-old C57 was kept in a constant temperature and humidity environment, with 12 hours of brightness/darkness a day and was free to drink and eat. The mice were deliberately separated into 2 groups: the control group and the model group. BLM was intraperitoneally injected at 4 mg/kg, while the control group was added with the same amount of normal saline. After 28 days, the mice were sacrificed, and their lung tissues were collected. All research involving animals must be approved and supervised by the Laboratory Animal Welfare and Ethics Committee of the Army Medical University. The HE and Masson staining showed that BLM induced pulmonary fibrosis in mice. And pulmonary fibrosis human samples come from the pathology department of the hospital, and all samples follow the application of human ethics and are accepted by the review of the clinical ethics committee of Daping Hospital.

### 2.5. Immunohistochemical Staining and Analysis

Immunohistochemical staining was performed according to standard procedures. Sections were stained with mouse monoclonal METTL3 antibody (Cat No: 67733-1-Ig, 1 : 400, Proteintech, Wuhan, China) overnight at 4°C and then rinsed with PBS and incubated with its associated HRP-conjugated secondary antibody (MXB biotechnologies, Cat No. Kit-5030, Fujian, China) for 30 min at room temperature. The sections were washed with PBS and developed with DAB, and then the sections were dyed with hematoxylin for nuclear staining. Positive staining is detected as brown and observed by an Olympus upright microscope.

### 2.6. Masson Staining

Stain with Wiegert iron hematoxylin staining solution, then stain with acidic ethanol differentiation solution, blue solution back to blue, ponceau red magenta staining solution, and wash the sections with acetic acid working solution; after treatment with phosphomolybdic acid solution, stain with aniline blue. Solution counterstain, treat the slices with an acetic acid working solution until the slices do not come off blue, then observe with an Olympus upright microscope (Cat. No: G1345, Solarbio, Beijing, China).

## 3. Results

### 3.1. m6A Methylation Regulators Identification by Consensus Clustering

The m6A methylation regulators which were considered consensus clusters were constructed. The consensus clustering cumulative distribution function (CDF) for *k* = 2 to 9, the area under the CDF curve for *K* = 2 to 9 showed a change compared to Figures 1(a) and 1(b). According to the m6A methylation regulator expression, the *k* value was determined, the most obvious difference was *k* = 2 (Figure 1(c)). At *k* = 2, pulmonary fibrosis samples are divided into two subgroups: cluster 1 and cluster 2. We identified and labeled cluster 1 and cluster 2, and the tracking plot demonstrated the *k* = 2 to *k* = 10 (Figure 1(d)).

### 3.2. Pulmonary Fibrosis Were Associated with Categories Identified by Consensus Clustering

The protein-protein interaction among these m6a methylation regulators is analyzed to better explain the inner relationship among the 10 m6A methylation regulators. The protein-protein interaction network was constructed (Figure 2(b)), and the top 5 hub genes were listed by the ranking method, which are WTAP, YTHDC2, METTL14, YTHDF2, and METTL3 (Figure 2(c)). According to the results, the expression of METTL3 was significantly associated with METTL14, WTAP, YTHDC2, METTL14, and YTHDF2 (Figure 2(d)). Cluster 1 and cluster 2 groups have been compared in the transcriptional profile by principal component analysis (PCA). There is an obvious distinction between cluster 1 and cluster 2 (Figure 2(a)). These results point out that these two subgroups identified by consensus clustering were associated with pulmonary fibrosis. Logistic regression demonstrated strong correlations with m6A methylation regulators in pulmonary fibrosis (Table 1).

### 3.3. Predictive Evaluation Point Out That Strong Correlation with Clinicopathological Features in Pulmonary Fibrosis

The relationships between the m6A methylation regulators and clinicopathological features was shown by heatmap in pulmonary fibrosis (Figure 3(a)). The data indicated that there were significant differences between the health and fibrosis disease groups in terms concerning patient's status, indicating that biomarkers calculated by signatures can accurately predict the occurrence of fibrosis in patients (Figure 3(b)). Then, we used another GEO (GSE110147) data set for verification and found that METTL3 can still effectively predict the occurrence of pulmonary fibrosis in fibrotic tissue (Figures 3(c) and 3(d)).

To verify the correctness of this model, we searched for 17 columns of human pulmonary fibrosis samples and 3 columns of normal lung tissue samples and performed immunohistochemical staining. The results indicated that METTL3 was lower expressed in pulmonary fibrosis tissues (Figure 4(a)), and low expression of METL3 was also observed in pulmonary fibrosis induced by bleomycin (Figure 4(b)). In conclusion, the M6A methyltransferase METTL3 may be used as a molecular marker and a potential therapeutic target for the occurrence and development of pulmonary fibrosis.

## 4. Discussion

While the last two decades have seen impressive progress made in biomarker discovery, many of the alveolar lavage fluid and serum protein biomarkers discriminate pulmonary fibrosis from healthy controls. Despite the considerable work performed in this arena, test performance for individual biomarkers has generally been insufficient to justify their incorporation into clinical practice.

At present, the main biomarkers of pulmonary fibrosis are as follows: MMP-9 [21], KL-6 [22], S100A6 [23], and MMP7 [21], but as we know, pulmonary fibrosis is an extremely complex disease, and a single biomarker is an inaccurate representation of pulmonary fibrosis status. Therefore, finding more pulmonary fibrosis markers has a deeper meaning.

Previous studies have revealed that m6A methylation regulators are associated with RNA translation disorders in cancer occurrence and development [24, 25]. However, more and more evidence shows that this process not only occurs in tumors but also occurs in various diseases [26]. We analyzed the expression of m6A methylation regulators in pulmonary fibrosis to determine whether the expression of m6A methylation regulators can be regarded as a diagnosis maker, which is a key point for early diagnosis and treatment of pulmonary fibrosis [27]. The m6A methylation regulator METTL3 as a prediction maker has been addressed thoroughly in pulmonary fibrosis. Next, it could be designed with related drugs for METTL3, which may be used as a new treatment target for pulmonary fibrosis.

The m6A methylation regulators was found in this study to construct the pulmonary fibrosis biomarkers. The risk signature based on the minimum criteria based on METTL3 has been built, and the coefficients based on the logistic algorithm were used to calculate the odds ratio. The ROC curve demonstrated that there are m6A methylation regulators METTL3 in pulmonary fibrosis and can be used as a useful tool for developing novel therapeutic targets for pulmonary fibrosis diagnosis.

## 5. Conclusions

In this study, we showed that the expression of m6A methylation regulators was associated with pulmonary fibrosis. There are two pulmonary fibrosis groups, which were calculated by consensus clustering based on the expression of m6A methylation regulators. Also, a biomarker signature was constructed with the selected m6A methylation regulators. And verified on biological samples, the results showed that METTL3 was significantly reduced in fibrosis patients and in Bleomycin-induced pulmonary fibrosis models. It is shown that METTL3 may be used as a molecular marker for the treatment and prognosis of pulmonary fibrosis.

## Figures and Tables

**Figure 1:** Identify consensus clusters by m6A methylation modulators. (a) CDF (consensus clustering cumulative distribution function), *k* = 2 to 9. (b) *k* = 2 to 9, the area under CDF curve was relative change and the consensus clustering matrix when *k* = 2. (d) The tracking plot for *k* = 2 to *k* = 10.

**Figure 2:** Interaction among the m6A methylation regulators has been shown by the PPI (the protein-protein interaction) network. (a) PCA of the sequencing data profile in the pulmonary fibrosis data extracted from the GEO data set. (b) The PPI network shows the interaction among m6A methylation regulators in the online database. (c) 10 hub genes were demonstrated according to the online PPI network. (d) 10 m6A modification regulators analysis by the Spearman correlation.

**Figure 3:** The clinicopathological characteristics, ROC, and cluster subgroups. The heatmap demonstrates the expression level of the m6A methylation regulators in GSE33356 (a) and GSE110147 (c). ROC of GSE33356 (b) and GSE110147 (d) to show the risk of the pulmonary fibrosis inner relationship with m6A methylation regulators.

**Figure 4:** Animal samples and human samples to verify the relationship between m6A methylation and pulmonary fibrosis (H&E 10X Masson 40X, IHC 20X).

**Table 1:** Logistic regression analysis value of each m6a methylation regulators.

Gene	*p* value	OR	Confidence interval	
			Upper 95%	Lower 95%
METTL14	0.010	0.224	0.072	0.697
METTL3	0.006	0.359	0.174	0.742
RBM15	0.811	1.139	0.394	3.291
WTAP	0.426	0.747	0.364	1.533
YTHDC1	0.212	0.608	0.279	1.327
YTHDC2	0.011	0.263	0.094	0.737
YTHDF1	0.117	2.633	0.784	8.841
YTHDF2	0.535	0.759	0.318	1.812
ALKBH5	0.047	3.022	1.017	8.978
FTO	0.354	0.674	0.293	1.551

## Data Availability

All the data were obtained from the GEO dataset and can be found on NCBI.
